# KRAS activation in gastric cancer stem-like cells promotes tumor angiogenesis and metastasis

**DOI:** 10.1186/s12885-023-11170-0

**Published:** 2023-07-22

**Authors:** Changhwan Yoon, Jun Lu, Yukyung Jun, Yun-Suhk Suh, Bang-Jin Kim, Jacob E. Till, Jong Hyun Kim, Sara H. Keshavjee, Sandra Ryeom, Sam S. Yoon

**Affiliations:** 1 Department of Surgery, Columbia University Irving Medical Center, Milstein Hospital Building 7-002, 177 Fort Washington Avenue, New York, NY 10032 USA; 2 Department of Gastric Surgery, Fujian Medical University Union Hospital, Fuzhou, Fujian China; 3 Center for Supercomputing Applications, Korea Institute of Science and Technology Information, Division of National, SupercomputingDaejeon, Korea; 4 Department of Surgery, Seoul National University, Bundang Hospital, Seongnam, Korea; 5 Department of Surgery, Seoul National University College of Medicine, Seoul, Korea; 6 Department of Cancer Biology, Perelman School of Medicine, University of Pennsylvania, Philadelphia, PA USA; 7 Department of Biological Science, Hyupsung University, Hwasung-Si, Republic of Korea

**Keywords:** Gastric adenocarcinoma, KRAS, Epithelial-to-mesenchymal transition, Cancer stem cells

## Abstract

Our previous work showed that KRAS activation in gastric cancer cells leads to activation of an epithelial-to-mesenchymal transition (EMT) program and generation of cancer stem-like cells (CSCs). Here we analyze how this KRAS activation in gastric CSCs promotes tumor angiogenesis and metastasis. Gastric cancer CSCs were found to secrete pro-angiogenic factors such as vascular endothelial growth factor A (VEGF-A), and inhibition of KRAS markedly reduced secretion of these factors. In a genetically engineered mouse model, gastric tumorigenesis was markedly attenuated when both KRAS and VEGF-A signaling were blocked. In orthotropic implant and experimental metastasis models, silencing of KRAS and VEGF-A using shRNA in gastric CSCs abrogated primary tumor formation, lymph node metastasis, and lung metastasis far greater than individual silencing of KRAS or VEGF-A. Analysis of gastric cancer patient samples using RNA sequencing revealed a clear association between high expression of the gastric CSC marker CD44 and expression of both KRAS and VEGF-A, and high CD44 and VEGF-A expression predicted worse overall survival. In conclusion, KRAS activation in gastric CSCs enhances secretion of pro-angiogenic factors and promotes tumor progression and metastasis.

**Supplementary Information:**

The online version contains supplementary material available at 10.1186/s12885-023-11170-0.

## Background

Worldwide, there are over one million new gastric cancer cases and nearly 800,000 gastric cancer deaths per year, and thus gastric cancer accounts for almost 10% of all cancer deaths [1]. Gastric adenocarcinomas (GAs) comprise the vast majority of gastric cancers, and most patients with GA present with locally advanced or metastatic disease. The response rate of GA to chemotherapy can be 50% or greater, but nearly all patients develop chemotherapy resistance, and median survival is extended only to about one year [2]. Thus, there is an urgent need for new and more effective therapies.

In the Cancer Genome Atlas (TCGA) study of GA, genes encoding the Receptor Tyrosine Kinase (RTK)-RAS signaling pathway were altered in 60% of GAs [3]. The RAS family of proteins in humans includes KRAS, HRAS, and NRAS [4], and *KRAS* is specifically amplified or mutated in 17% of GAs [3]. Upon stimulation by upstream receptors, KRAS recruits RAF to the cell membrane where it promotes RAF dimerization and activation. Activated RAF phosphorylates and activates MEK, and activated MEK in turn phosphorylates and activates ERK.

We previously found that oncogenic *Kras* can increase gastric tumorigenesis and metastasis in a genetically engineered mouse model [5]. In GA driven by *Cdh1* loss and *Trp53* loss in gastric parietal cells, 69% of mice developed diffuse-type GA that metastasized to lymph nodes at one year [6]. Combining *Cdh1* loss and *Trp53* loss with oncogenic *Kras* (*Kras*^*G12D*^) increased the penetrance of GA to 100% and reduced survival to 76days. In these mice, both intestinal and diffuse primary tumors were observed throughout the stomach, as well as lymph node, lung, and liver metastases. In a subsequent study, we demonstrated that KRAS activation promotes epithelial to mesenchymal transition (EMT) and acquisition of cancer stem-like cell (CSC) phenotypes, including metastatic potential and chemoresistance [7]. Levels of KRAS and levels of KRAS activation in numerous gastric cancer cells lines grown as monolayers and as spheroids were significantly increased in gastric cancer cells grown as spheroids vs. monolayers. CD44 is a marker of gastric cancer stem-like cells. CD44( +) cells exhibited significantly higher levels of KRAS signaling activation compared to CD44(-) cells. However, the exact mechanism by which metastasis was enhanced was not specifically elucidated.

Angiogenesis, or new blood vessel formation, is a vital process in the progression and metastasis of solid tumors, including GA [8]. Tumors induce angiogenesis by secreting pro-angiogenic molecules such as vascular endothelial growth factor A (VEGF-A), and VEGF-A inhibition has become a common therapeutic strategy for many cancers [9]. Several drugs targeting the VEGF-A pathway have been approved for clinical use in selected solid tumors, and several anti-VEGF-A strategies have been examined for GA. Two international phase III trials examined ramucirumab, an antibody targeting the primary receptor for VEGF-A, VEGFR-2, as second line therapy for advanced GA and found a survival benefit both as single agent therapy and when combined with chemotherapy [10, 11].

In this study, we hypothesized that KRAS signaling in gastric CSCs promotes the secretion of pro-angiogenic factors that would enhance primary tumor formation and metastasis.

## Materials and method

### Human cell lines and reagents

AGS (RRID CVCL_0139: KRAS^G12D^) and NCI-N87 (RRID CVCL_1603:KARS^WT^) subsequently referred to as N87 are Lauren intestinal-type GA cell lines, and MKN-45 (PRID CVCL_0434: KRAS^WT^), KATOIII (RRID CVCL_0371:KRAS^WT^) and SNU-668 (RRID CVCL_5081:KRAS^Q61K^) are Lauren diffuse-type GA cell line. AGS, MKN-45 and N87 cells were obtained from the America Type Culture Collection (ATCC). KATOIII and SNU-668 cells were obtained from the Korean Cell Line Bank (KCLB). Cancer cell lines were actively passaged for less than 6months from the time that they were received from the ATCC or KCLB, and United Kingdom Co-ordinating Committee on Cancer Research (UKCCCR) guidelines were followed [12]. KATOIII cells were maintained in DMEM, and the other GA cell lines were maintained in RPMI 1640. All media were supplemented with 10% FBS, 100 U/mL penicillin and 100 mg/mL streptomycin, and L-glutamine 2mmol/L ("regular media"). Human umbilical vein endothelial cells (HUVEC) were obtained from Lonza (Basel, Switzerland) and used within 8 passages. All endothelial cells were grown in EGM-2-MV media (Lonza). Mouse Primary Vein Endothelial Cells (MVEC; Cell biologics, C57-6009) were maintained with Endothelial Cell Medium /w Kit (Cell Biologics, M1168).

Reagents were purchased from the following sources: XenoLight D-Luciferin, PerkinElmer Inc. (#122,799); MEK inhibitor, Santa Cruz (sc-364412A); Matrigel, BD Bioscience (Cat. 354,248); B27, Sigma-Aldrich (0080085SA); N2, Thermo Fisher Scientific (A13707-01); N-acetylcysteine, Sigma-Aldrich (A9145); Epidermal growth factor (EGF), Sigma Aldrich (E9644); Fibroblast growth factor-basic (FGF-Basic), Sigma Aldrich (341,583); Gastrin I, Sigma Aldrich (G9145); Nicotinamide, Sigma Aldrich (N0636), Y-27632, Sigma Aldrich (Y0503); SB202190, Sigma Aldrich (S7067); Prostaglandin E2, Tocris Bioscience (#2296); Recombinant Rspondin 1, PeproTech (120–38); mNoggin, PeproTech (250–38); Wnt3A, R&D Systems (5036-WIN); FGF-10, PeproTech (100–26); A83-01, R&D Systems (#2939); Recombinant human-VEGF-A, R&D Systems (293-VE-010), FGF-2, R&D Systems (233-FB-010).

### Spheroid generation

Cells were resuspended in spheroid media comprised of DMEM/F12 containing epidermal growth factor (EGF), basic fibroblast growth factor (bFGF), N-2 supplement, and B27 and then plated on ultra-low attachment culture dishes (Corning Life Sciences). Spheroids were collected after 5–7days except when noted otherwise. Proteins were extracted for analysis, or cells were dissociated with Accutase and used for other experiments. Spheroid growth was quantified as the average number of spheroids > 50–100μm in diameter among 5 fields after image processing using Imaris 7.6 (Bitplane).

### Mouse tumor-derived organoids and cell lines

The Tcon3077 and Tcon3944 gastric tumors were harvested from Tcon mice (see below), and organoids were generated and maintained as previously described [13]. Tcon3077 and Tcon3944 cell lines were also generated from Tcon tumors. Tcon cell lines were maintained in DMEM supplemented with 10% FBS, 100 U/mL penicillin and 100mg/mL streptomycin, and L-glutamine 2mmol/L ("regular media").

### Western blot analysis

Proteins were extracted by collecting cells in RIPA buffer (Sigma-Aldrich) containing Complete Protease Inhibitor Cocktail (Roche), and protein concentration was determined using the Bio-Rad Protein Assay (Bio-Rad). Proteins were detected using the following antibodies: KRAS (sc-30) from Santa Cruz.; VEGF-A (ab46154, sc-7269) from Abcam and Santa Cruz; and β-actin (A5441) from Sigma.

### Lentiviral transduction

VEGF-A was silenced via lentiviral transduction of mouse VEGF shRNA (sc-36815-V; Santa Cruz Biotechnology). KRAS was silenced via lentiviral transduction of human or mouse KRAS shRNA (sc-36815-V, sc-43876-V; Santa Cruz Biotechnology). Lentiviral transduction of a scramble shRNA (sc-108080; Santa Cruz) was used as a control. Luciferase (firefly) lentivirus (FCT005, Kerafast, Inc.) was transduced following the manufacturer’s protocol. Maximal knockdown of genes occurred 72–96h after transduction.

### Angiogenesis antibody arrays

To generate condition media, we used DMEM without FBS for monolayer cells and DMEM witih B27 and N2 for spheroids (basal media). The relative levels of human and mouse angiogenesis-related proteins in GA cells grown as monolayers and as spheroids were measured using the Proteome Profiler Human Angiogenesis Array Kit and Proteome Profiler Mouse Angiogenesis Array Kit (ARY007, ARY015, R&D Systems Inc.) following the manufacturer’s protocol. The results were analyzed with ImageJ software.

### Human and mouse endothelial cell tube formation assay

Tube formation assays were performed in Matrigel-coated (BD Biosciences) 24-well plates. To generate condition media, we used DMEM without FBS for monolayer cells and DMEM witih B27 and N2 for spheroids (basal media). Conditioned media from GA cells treated with control, KRAS and/or VEGF-A shRNA were collected after 3days. After HUVEC (3 × 10^4^) and MVEC (3 × 10^4^) were seeded on the 24 wells in 12h, 300 μL of conditioned medium from cancer cells were replaced. Images were taken using a bright-field microscope at 100 × magnification, and the total length of completed tubule structures was quantified.

### Gastric cancer mouse models

The study was performed in accordance with the relevant guidelines and regulations. All animal protocols were approved by the Institutional Animal Care and Use Ethics Committee, Columbia University. This research was in accordance with ARRIVE quidelines. Tcon mice were generated by cross breeding as previously described [5]. Treatment of Tcon mice with a MEK inhibitor (PD0325901, APExBIO) was initiated in 4-week-old mice (*n* = 7 per group). The drug was administered ad libitum in the mouse chow (Purina 5010) at 7mg/kg (incorporation by Research Diets Inc). The same mouse chow without drug was used as the control. DC101 (50–562-188, Bio X Cell) 20mg/kg ip or control IgG antibody 20mg/kg ip was also initiated in 4-week-old mice. At 10weeks, 2 mice from each group were sacrificed and tumors were harvested. Stomachs were fixed in 10% buffered formalin for 24h, embedded in paraffin, and processed into 5µm sections.

For orthotropic intra-gastric injection mouse models, anesthesized mice were injected with 1 × 10^5^ CD44( +) cells in 100 ul /HBSS into the gastric wall via a laparotomy incision. At 8, 10, 12, and 15weeks after tumor cell injection, mice (n = 7 per group) were intraperitoneally injected with 100 µL D-luciferin solution (150 mg/kg, #122,799, Perkin Elmer), anesthesized with 2% isoflurane, and imaged in a Xenogen IVIS 200 (PerkinElmer) after 5min according to the manufacture's protocol. To harvest the tumors, 2 mice in each group were sacrificed at 12 weeks, stomachs were harvested and processed as above.

### Lung, liver, and lymph node metastasis models

To generate experimental lung metastases, mice were injected via the tail vein with 5 × 10^4^ CD44( +), CD44(-), or unsorted Tcon3077 cells (*n* = 6 per group). Mince were sacrificed at 3.5weeks. Lungs of all mice were fixed in 10% buffered formalin for 24h, embedded in paraffin, and processed into 10m sections. For each mouse lung, 10 sections were examined by H&E staining for lungs metastases. In a subsequent experiment, 5 X10^4^ CD44( +) cell stably transduced with control shRNA, KRAS shRNA, VEGF-A shRNA, or both KRAS and VEGF-A shRNA were injected into the tail vein of mice (*n* = 7 per group). At 3.5weeks after tumor cell injection, mice were intraperitoneally injected with 100 μL D-luciferin solution (150mg/kg, #122,799, Perkin Elmer), anesthetized with 2% isoflurane, and imaged in a Xenogen IVIS 200 (PerkinElmer) after 5min according to the manufacture's protocol. Mice were then sacrificed, and lungs were harvested.

To generate experimental liver metastases, 5 × 10^4^ Tcon3077 CD44( +) cells were injected into the spleen (*n* = 6 per group). At 2, 3, and 4weeks after tumor cell injection, mice were intraperitoneally injected with 100 μL D-luciferin solution (150mg/kg, #122,799, Perkin Elmer), anesthetized with 2% isoflurane, and imaged in a Xenogen IVIS 200 after 5min according to the manufacture's protocol. Mice were sacrificed at 4weeks, and livers and spleens were harvested. Livers and spleens of all mice were fixed in 10% buffered formalin for 24h, embedded in paraffin, and processed into 10μm sections. For each mouse liver and lung, 10 sections were examined.

To generate lymph node metastases, 5 × 10^4^ Tcon3077 CD44( +) cells grown from cells were injected into the foot-pads of mice on day 0 (*n* = 6 per group). Following sacrifice at 4weeks, enlarged inguinal lymph nodes were harvested, fixed in 10% buffered formalin for 24h, embedded in paraffin, and processed into 10μm sections.

### Immunohistochemistry (IHC)

Immunohistochemistry was performed for patient and mouse tumor samples using the following primary antibodies: CD31 (MA5-13,188; Thermo Fisher Scientific), CD44 (NBP1-31,488; NOVUS Biological USA), p-MEK1/2 (#9154; Cell signaling), YFP (MBS833304; MYBIOSource), p-ERK1/2 (#9101; Cell signaling), VEGF-A (sc-7269; Santa Cruz), and LYVE-1 (AF2089, AF2125; R&D system).

#### Validation in independent patient cohorts

RNA-seq data of paired normal and tumor samples for 83 GAs from Jun et al. were used for independent validation [14]. We performed hierarchical clustering using ComplexHeatmap v2.9.3 [15] with log_2_ fold-change values of three genes (KRAS, VEGFA, and CD44), and divided patients into three subgroups based on CD44 expression. Fisher’s exact and Chi-squared tests were performed to evaluate differences between subgroups. Gene set enrichment analysis was used to identify overrepresented biological functions using Gene Set Enrichment Analysis (GSEA) [16]. We calculated the enrichment scores using gene sets from the MSigDB Hallmark collection (*n* = 50) [17].

#### Patient samples

Gastric tumors from surgically resected specimens were fixed in formalin, embedded in paraffin, and sectioned. GC sections or FMUUH patient tumor TMAs were deparaffinized prior to incubation with antibodies against human CD44 (NBP1-31,488; NOVUS Biological USA) and VEGF-A (sc-7269; Santa Cruz) in a solution of PBS with 1% BSA and 0.1% Triton X-100 at 4 C overnight according to standard protocols as previously described. The intensity of staining for CD44 and VEGF-A was scored as 0 to 3. The proportion of positively stained cells was scored as follows: ≤ 5% positive cells, 0; 6 to 25% positive cells, 1; 26 to 50% positive cells, 2; ≥ 51% positive cells, 3. To obtain an IHC score that considers the IHC signal intensity and the frequency of positive cells, the intensity score was multiplied by the percentage score. Composite scores less than 3 were defined as low expression and scores of 4 or higher as high expression.

#### Statistical analysis

Data are represented as mean ± standard deviation unless otherwise noted. Statistical analyses were performed using GraphPad9. P values were calculated using Student’s t-test, except for comparisons between more than two groups, in which case treatment groups were compared to controls using one-way ANOVA with Bonferroni adjustment for multiple comparisons.

For analyses of patient data, categorical variables were analyzed using χ^2^ or Fisher’s exact test. Overall survival curves were plotted using Kaplan–Meier methods and compared by the log-rank test. Cox proportional hazards regression modeling was used to examine the relationship between CD44 and VEGF-A expression and survival, while controlling for confounding covariates. Analyses were performed using IBM SPSS software for Windows version 21 (IBM). A *p* value < 0.05 was considered statistically significant.

## Results

### Conditioned media from gastric cancer spheroid cells promotes angiogenesis

We have previously described a genetically engineered mouse model of GA driven by loss of *Trp53*, loss of *Cdh1*, and addition of oncogenic *Kras*^*G12D*^ in gastric parietal cells [5]. These triple conditional or Tcon mice developed both intestinal and diffuse type GAs with 100% penetrance and metastases to lymph nodes, lung, and liver. We generated tumor-derived organoids and cell lines from two tumors from Tcon mice and labelled them Tcon3077 and Tcon3944.

Growth of tumor cells as spheroids enriches for cancer stem-like cells (CSCs) [18]. We first harvested conditioned media from Tcon3944 cells grown as monolayer cells and as spheroids, and applied the conditioned media to mouse vein endothelial cells (MVEC) in a tube formation assay. Conditioned media from Tcon3944 spheroid cells led do a 2.2-fold increase in tube formation compared to conditioned media from Tcon3944 monolayers cells (Fig. 1A). Similar results were seen with conditioned media from Tcon3077 cells (data not shown). We next examined human umbilical vein endothelial cell (HUVEC) tube formation in conditioned media from four human GA cell lines (AGS, MKN-45, SNU668, and KATOIII) grown as monolayers or as spheroids. Conditioned media from spheroid cells led to a 1.9–4.3-fold increase in tube formation compared to conditioned media from monolayer cells (Fig. 1B).

**Fig. 1:** Conditioned media from GA spheroid cells promotes angiogenesis. **A** Tube formation assay using Mouse Primary Vein Endothelial Cells (MVECs) in conditioned medium from Tcon3944 mouse GA cells grown as monolayers and spheroids with basal media devoid. **B** Tube formation assay using Human Umbilical Vein Endothelial Cells (HUVECs) in conditioned medium from human GA cells grown as monolayers and spheroids. **C** Western blot for KRAS in spheroid cells transduced with KRAS shRNA (sh.KRAS) and control scramble shRNA (sh.Scr). β-actin was used as a loading control (Original version in Suppl. Figs. S5A, B). **D**-**E** Tube formation assay of MVECs or HUVECs in conditioned media from spheroids transduced with sh.KRAS and sh.Scr. Scale bar, 50m. Bars represent standard deviation. *p < 0.05 compared to control

To determine if KRAS promotes secretion of angiogenic factors in GA spheroid cells, we knocked down KRAS using shRNA. The knockdown efficiency of KRAS in all GA cell lines was confirmed by Western blot analysis (Fig. 1C, Suppl. Figs. S5A, B). KRAS knockdown in Tcon3944 spheroid cells reduced the ability of conditioned media to promote MVEC tube formation by 86.3% (Fig. 1D). Similar results were found when KRAS was knocked down in Tcon3077 spheroid cells (data not shown) and in spheroid cells from the four human GA cell lines, with decreases in HUVEC tube formation of 75–91% (Fig. 1E). These data suggest that KRAS activation in GA spheroid cells promotes secretion of pro-angiogenic factors.

### KRAS promotes GA spheroid cell secretion of VEGF-A, FGF-2, and/or EGF

To determine which pro-angiogenic factors were being secreted, we collected conditioned media from Tcon3944 cells grown as monolayers and as spheroids and examined for secreted angiogenic factors using the Proteome Profiler Mouse Angiogenesis Array kit. The four angiogenic factors secreted most by Tcon3944 spheroid cells relative to monolayer cells were FGF-2, IL-1α, EGF, and VEGF-A (spheroid secretion 5.7–13.5-fold higher than monolayer secretion) (Fig. 2A). KRAS shRNA knockdown in Tcon3944 spheroid cells led to 72–81% reductions in the secretion of these factors, including an 80% reduction in VEGF-A secretion (Fig. 2B). The angiogenic secretomes of SNU668 human GA cells grown as spheroids and as monolayers differed somewhat from that of Tcon3944 cells. Secretion of EGF, Amphiregulin, and VEGF were upregulated 10.8–36.6-fold (Fig. 2C). KRAS shRNA in SNU668 spheroid cells led to 49–80% reductions in secretion of these angiogenic factors, including an 80% reduction in VEGF-A secretion (Fig. 2D). The angiogenic factors EGF and FGF-2 were also secreted at increased levels by AGS and MKN-45 spheroid cells compared to monolayers cells (Suppl. Figs. S1A, B). VEGF-A secretion was only 2.2–3.1-fold higher. However, for all five cells lines, KRAS shRNA dramatically reduced VEGF-A secretion between 50–90% (Figs. 2B, D, Suppl. Figs. S1C, D).

**Fig. 2:** KRAS promotes GA spheroid cell secretion of VEGF-A, FGF-2, and/or EGF. Graphs showing levels of secreted angiogenic factors into basal media devoid of supplements from Tcon3944 monolayer cells and spheroids **A** from Tcon3944 spheroids transduced with KRAS shRNA (sh.KRAS) and control scramble shRNA (sh.Scr). **B** as determined by the Proteome Profiler Mouse Angiogenesis Array kit. Graphs showing levels of secreted angiogenic factors from SNU668 monolayer cells and spheroids **C** and from SNU668 spheroids transduced with sh.KRAS and sh.Scr **D** as determined by the Proteome Profiler Human Angiogenesis Array kit. **E** Graph of tube formation with conditioned media from AGS and MKN-45 spheroids treated with sh.KRAS, sh.Scr, recombinant EGF (rEGF), recombinant VEGF-A (rVEGF-A), or recombinant FGF-2 (rFGF-2). Bars represent standard deviation. *p < 0.05 compared to control

To confirm that VEGF-A, FGF-2, and/or EGF were responsible for promoting tube formation, we again knocked down KRAS in AGS and MKN-45 spheroid cells and applied the conditioned media supplemented with recombinant VEGF-A, FGF-2, or EGF to HUVEC in a tube formation assay. The addition of these pro-angiogenic factors partially restored tube formation, with recombinant VEGF-A having the most significant effect (Fig. 2E). These data confirm that KRAS activation promotes secretion of pro-angiogenic factors including VEGF-A in GA spheroid cells.

### RTK/KRAS and VEGF-A/VEGFR-2 in GA organoid cells combine to promote primary tumor growth

To examine the role of the KRAS and VEGF-A in tumor-derived organoid formation, we knocked down KRAS, VEGF-A, or both in Tcon3077 cells and grew them as organoids. Western blot analysis confirmed stable KRAS and/or VEGF-A knockdown by shRNA in Tcon3077 organoids (Suppl. Figs. S1E, S6A). KRAS shRNA attenuated organoid growth, but VEGF-A shRNA did not (Fig. 3A). In addition, expression of the CSC marker CD44 in Tcon3077 organoids was reduced by KRAS shRNA but not by VEGF-A shRNA. (Fig. 3B).

**Fig. 3:** RTK/KRAS and VEGF-A/VEGFR-2 inhibition block GA progression in Tcon mice. **A** Representative H&E photos of Tcon3077 organoids following transduction with VEGF-A shRNA (sh.VEGF-A) and/or KRAS shRNA (sh.KRAS) or control scramble shRNA. Graph showing number of organoids greater than 100m. **B** Immunofluorescence (IF) photos showing CD44 (green) and cell nuclei (DAPI). Graph showing the percent of DAPI positive cells with expression of the cancer stem cell maker, CD44 in transduced Tcon3077 organoids. **C** Survival curve of Tcon mice treated with an oral MEK inhibitor, DC101, both MEK inhibitor and DC101, or control (*n* = 5–7 per group). **D** Representative photos of H&E slides for stomach mouse tumors. **E**–**F** IHC and graphs for CD44 and CD31 expression in mouse stomach tumors. Bars represent standard deviation. *p < 0.05 compared to control. **p < 0.05 compared to all other groups

We previously inhibited RTK/KRAS signaling in Tcon mice by treating with a MEK inhibitor starting at 4weeks of age, and median survival increased from 76 to 95 days [5]. DC101 is a neutralizing antibody for VEGFR-2, the primary receptor for VEGF-A [19]. We next examined the combination of VEGF-A inhibition and MEK inhibition in Tcon mice (*n* = 7 per group). MEK inhibition alone increased median survival by 23 days, DC101 increased median survival by 45 days, and combination therapy increased median survival by 91 days (Fig. 3C). Two mice in each group were sacrificed at 10 weeks of age, and 3 tumors in each stomach were examined. Inhibition of both MEK and VEGF-A at this time point led to smaller and earlier stage stomach tumors (Fig. 3D), decreased expression of the CSC marker CD44 (Fig. 3E, Suppl. Fig. S2A), and decreased microvessel density (Fig. 3F, Suppl. Fig. S2B) compared to MEK inhibition alone or VEGF-A inhibition alone.

The effects of RTK-RAS and VEGF-A/VEGFR-2 inhibition were next examined in an orthotropic model of GA. CD44 + Tcon3077 cells were isolated by FACS and then stably transduced with lentiviral shRNA vectors to knockdown KRAS, VEGF-A, or both (Fig. 4A, Suppl. Fig. S6B). The lentiviral shRNA vectors also transduced the luciferase reporter gene. Stably transduced CD44 + Tcon3077 cells were grown as organoids and injected into the gastric wall of syngeneic mice (*n* = 7 per group) and bioluminescence imaging using the Xenogen IVIS system was performed at 8, 10, 12, and 15 weeks. At 10 weeks, tumor bioluminescence was decreased by 39% with KRAS knockdown, 44% with VEGF-A knockdown, and 96% with combined KRAS and VEGF-A knockdown (Fig. 4B). Two mice were sacrificed at 12 weeks and stomach were analyzed. In this orthotopic model, mice generally develop a single tumor at the injection site. By gross inspection, tumors from control organoid cells were large, tumors from organoid cells with knockdown of KRAS or VEGF-A were intermediate in size, and tumors from organoid cells with knockdown of both KRAS and VEGF-A were hard to distinguish (Fig. 4C). Given only two tumors were analyzed for each group, we increased the number of sections analyzed per tumor from 3 to 5. Following H&E staining, tumors were identified in all 4 groups, but tumors from organoid cells with knockdown of both KRAS and VEGF-A were small and early stage (Fig. 4C, Suppl. Fig. S2C). Tumors were then stained by immunofluorescence for CD44, CD31, and phosphorylated MEK (Fig. 4D). Knockdown of KRAS or VEGF-A led to reduced expression of CD44, CD31, and phosphorylated MEK by 36.7–61.5%, while knockdown of both KRAS and VEGF-A reduced expression of these proteins by 94.1–95.6%. Median survival of mice was 66 days, 85 days, 91 days, and 121 days for tumors with no knockdown, knockdown of KRAS, knockdown of VEGF-A, and knockdown of both KRAS and VEGF-A, respectively (Fig. 4E).

**Fig. 4:** Inhibition of RTK-RAS and VEGF-A/VEGFR2 blocks tumorigenesis in an orthotropic model of GA. **A** Western blot analysis for KRAS, VEGF-A and β-actin in CD44( +) Tcon3077 cells stably transduced with KRAS shRNA (sh.KRAS), VEGF-A shRNA (sh.VEGF-A) and/or control scramble shRNA (Original version in Suppl. Figs. S6B-C). **B** IVIS images 10 weeks after intra-gastric injection of CD44( +) Tcon3077 cells transduced with sh.KRAS and/or sh.VEGF-A. Graph showing bioluminescence for each group. **C** Representative gross photos and H&E slides of stomach tumors in mice sacrificed at 12 weeks. **D** IF images of gastric tumors stained for CD44 (red), CD31 (white), and p-MEK1/2 (green). Graphs showing number of positive cells. **E** Survival curve of 4 groups of mice. Dashed line represents time of sacrifice (12weeks) of two mice for stomach tissue analysis. Bars represent standard deviation. *p < 0.05 compared to control. **p < 0.05 compared to all other groups

### RTK/KRAS and VEGF-A/VEGFR-2 in CD44( +) GA cells promotes metastasis

GA metastasizes to lymph nodes, liver, and lung. We examined the role of KRAS and VEGF-A in promoting metastases using experimental metastasis models. Tcon3077 cells were FACS sorted into CD44( +) and CD44(-) cells, and experimental lung metastases were generated by injecting CD44( +), CD44(-), and unsorted cells into the tail veins of syngeneic mice (n = 6 per group). Based on our previously published paper on CD44 expression in gastric cancer cells, the proportion of CD44-expressing cells in unsorted cells is less than 1% of the total cell population [18]. Mice were sacrificed 3.5 weeks after tumor cell injection, and lungs were examined by H&E staining. CD44( +) cells formed significantly more lung metastases than CD44(-) or unsorted cells (Fig. 5A). In a subsequent experiment, Tcon3077 CD44( +) cells were stably transduced with KRAS shRNA, VEGF-A shRNA, or both, and injected into the tail vein of syngeneic mice to form experimental lung metastases (*n* = 7 per group). At 3.5 weeks, bioluminescence imaging was performed, mice were sacrificed, and lungs were analyzed. Knockdown of KRAS or VEGF-A led to a 45–48% reduction in bioluminescence compared to controls, while knockdown of both KRAS and VEGF-A led to an 86% reduction (Fig. 5B, Suppl. Fig. S2D). H&E staining and YFP immunofluorescence revealed large lung metastases in control mice, smaller lung metastases in mice injected with cells with KRAS or VEGF-A knockdown, and only a few microscopic metastases in mice injected with cells with both KRAS and VEGF-A knockdown (Fig. 5C). Next VEGF-A immunohistochemistry and VEGF-A/CD31/CD44 triple immunofluorescence were performed on harvested lungs, and VEGF-A, CD31, and CD44 expression were all dramatically reduced in mice injected with cells with both KRAS and VEGF-A knockdown (Fig. 5D).

**Fig. 5:** RTK/KRAS and VEGF-A/VEGFR-2 inhibition CD44( +) GA cells blocks metastasis. **A** Representative H&E photos of mouse lungs 3.5 weeks after tail vein injection of CD44( +), CD44(-), and unsorted Tcon3077 cells. Graph showing number of metastases > 100m per field for each group. **B** Graph showing bioluminescence after IVIS imaging of mouse lungs 3.5 weeks after tail vein injection of Tcon3077 cells stably transduced with KRAS shRNA, VEGF-A shRNA, or both. Scramble shRNA was used as a control. **C** H&E and IF photos (YFP, yellow; DAPI, blue) of mouse lungs. Graphs show number of metastatic foci > 100m per field and percent of YFP-positive cells. **D** H&E, VEGF-A IHC, and VEGF-A (green)/CD31 (white)/CD44 (red) IF. Graphs showing the percent of CD44, VEGF-A, and CD31-expressing cells. Bars represent standard deviation. *p < 0.05 compared to control. **p < 0.05 compared to all other groups

Next, the effect of VEGF-A and KRAS knockdown in Tcon3077 cells was assessed in an experimental lymph node metastasis model [20]. CD44( +) Tcon3077 cells stably transduced with KRAS shRNA and VEGF-A shRNA or control shRNA were inoculated into the footpads of mice (*n* = 6 per group). After 4 weeks, inguinal lymph nodes were assessed. Mice bearing tumors cells with KRAS and VEGF-A knockdown had inguinal node metastases that were significantly smaller than those of mice bearing control tumors (Suppl. Figs. S3A, B). Lymphatic vessel endothelial hyaluronan receptor 1 (LYVE 1) is a cell surface receptor on lymphatic endothelial cells that can be used as a lymphatic endothelial cell marker [21]. Node metastases from cells with knockdown of KRAS and VEGF-A also had 3.8-fold reduced expression of LYVE-1 and 4.9-fold reduced expression of CD44 compared to control node metastases as measured by immunofluorescence staining (Suppl. Fig. S3C).

### Expression of CD44, KRAS, AND VEGFA genes in GA patient tumors

We next analyzed expression of CD44, KRAS, and VEGF-A using RNA-sequencing data from paired tumor and adjacent normal tissue samples from 83 GA patients previously examined by Jun et al. [14]. Expression of CD44, KRAS, and VEGF-A were significantly upregulated in tumor tissues compared with adjacent normal tissues (Fig. 6A, Suppl. Fig. S4A). Hierarchical clustering of patients based on log2 fold-change values of these three genes showed that patients could be divided into three groups as defined by CD44 expression level: CD44 Low, CD44 Intermediate, and CD44 High (Fig. 6B) [15]. A significant association was observed between the CD44 Low cluster and upper tumor location, whereas the CD44 High cluster had significantly more lower tumor location (*p* = 0.0156). Of note, our CD44 High cluster was also enriched for the microsatellite instability (MSI) subtype in the Cancer Genome Atlas (TCGA) and ACRG classifications [22].

**Fig. 6:** Expression of CD44, KRAS, and VEGFA in GA patient tumors. **A** Gene expression of CD44, KRAS, and VEGF-A in gastric tumors compared to adjacent normal tissues. **B** Hierarchical clustering of gene expression in 83 patient tumors based on the log_2_ fold-change in gene expression in tumor compared to adjacent normal tissue. Clinical information, including tumor location, Lauren classification, TNM stage, and the molecular classifications by Splicing, ACRG, and TCGA methods are indicated for the three clusters defined by CD44 expression (low, intermediate, and high). **C** Box plots of KRAS and VEGFA expression in each CD44 patient cluster. **D** Kaplan–Meier overall survival curves stratified by expression of VEGF-A in the FMUUH cohort

We performed a functional gene set enrichment analysis (GSEA) that compared the transcriptome data of the CD44 Low and CD44 High clusters using the MSigDB Hallmark gene sets [16, 17]. We found that tumors in the CD44 High cluster were significantly enriched in cancer promoting pathways such as epithelial-mesenchymal transition (EMT), hypoxia, and KRAS signaling up (Suppl. Fig. S4B). Both KRAS and VEGF-A expression were significantly higher in the CD44 High cluster than in the CD44 Low cluster (Fig. 6C), and the expression levels of the two genes showed a significant positive correlation (Suppl. Fig. S4C).

We previously demonstrated that higher expression of CD44 and phosphorylated MEK (a marker of KRAS pathway activation) in GA patient tumors are poor prognostic factors for overall survival [23]. We next investigated the prognostic significance of CD44 and VEGF-A in 112 GA patients undergoing surgical resection at Fujian Medical University Union Hospital (FMUUH). The clinicopathological characteristics of these patients are shown in Supplemental Table 1. Tumor samples were stained by immunofluorescence for expression of CD44 and VEGF-A (Suppl. Fig. S4D). We confirmed that patients with higher levels of tumor CD44 expression had worse 5-year overall survival than patients with lower levels of tumor CD44 expression (Suppl. Fig. S4E). Moreover, we found high expression of VEGF-A was significantly associated with worse overall survival (Fig. 6D). The worst overall survival was seen in patients with tumors with high level of both CD44 and VEGF-A (Suppl. Fig. S4F).

## Discussion

GAs and other solid tumors need to induce angiogenesis, or new blood vessel formation, to expand and metastasize [8]. Solid tumors are comprised of heterogeneous cell populations, and thus it would not be surprising that some populations could induce tumor angiogenesis better than others. CSCs are a minority subset of tumor cells with the capacity for self-renewal and differentiation [24]. These CSCs may be the primary source of metastases [25]. In a prior study, we found that KRAS is upregulated in gastric CSCs and drives various phenotypes including EMT, chemotherapy resistance, and metastasis [7]. In this study, we find that KRAS in CSCs drives secretion of pro-angiogenic factors including VEGF-A. Inhibition of both KRAS and VEGF-A either genetically by RNA interference or pharmacologically using inhibitors or antibodies greatly attenuates primary tumor growth, lymph node metastasis, and distant metastasis. Analysis of human tumors using RNA sequencing and IHC reveals a high correlation between expression of the CSC marker CD44 and expression of KRAS and VEGF-A. Furthermore, high CD44 and high VEGF-A expression correlate with worse overall survival. These data indicate that dual targeting of KRAS and VEGF-A may be an effective strategy against GA, particularly in those patients having tumors with high levels of KRAS activation and VEGF-A secretion.

There is evidence from other investigators and our group that RTK-RAS signaling is important in the epithelial-to-mesenchymal transition (EMT), maintenance of gastric CSCs, and gastric tumorigenesis. Many of the phenotypic differences between CSCs and bulk tumor cells that lack stemness can be attributed to epigenetic changes caused by the EMT program [26]. This link between the passage through EMT and the acquisition of stem-like properties is vital for cancer cells in order to metastasize. Some evidence linking RTK-RAS signaling to EMT and CSCs comes from Yoon et al*.,* who treated *Runx3*^*−/−*^* p53*^*−/−*^ murine gastric epithelial cells with TGF-β1 to induce EMT and found an increase in the *EGFR/Ras* gene expression signature [27]. The addition of EGF or the increased expression of KRAS led to increased sphere formation and colony formation in soft agar, suggesting that the EGFR/Ras pathway is involved in the promotion of EMT to generate CSCs. Finally, Min et al*.* found that inhibition of KRAS activation using a MEK inhibitor inhibited dysplastic organoids derived from Mist1-Kras^G12D^ mouse stomach corpus [28].

The relationship between RTK-RAS activation and CSC function has not been extensively studied in GA, but several studies of other gastrointestinal tumors have found that mutated KRAS promotes the emergence of stemness traits [29]. In colorectal cancer, Blaj et al*.* found that high MAPK activity (downstream of KRAS signalling) promoted EMT and marked a progenitor cell subpopulation that served as the predominant source of growth in flank xenografts [30]. Also in colorectal cancer, Moon et al*.* showed that in cells carrying mutated APC, oncogenic KRAS increases expression of CSC markers (CD44, CD133, and CD166), spheroid formation, and the size of xenografts [31]. In pancreatic CSCs, inhibition of KRAS led to downregulation of JNK signaling and loss of self-renewal and tumor-initiating capacity [32]. In this study, we found that at least part of the ability of CSCs to form metastases is due to their increased expression of KRAS, which in turn promotes secretion of pro-angiogenic factors.

There are few studies examining the role of CSCs in promoting tumor angiogenesis or on the role of that oncogenic pathways play in this process. However, the association between KRAS and VEGF-A has been examined in some tumor types. A study of 204 patients with lung adenocarcinoma found that KRAS mutation was significantly associated with a high level of co-expression of VEGF-A, VEGFR-1 and VEGFR-2 [33]. Takahashi et al*.* found that combining MEK1/2 inhibition and VEGF-A inhibition led to synergistic inhibitory effects on tumor growth and angiogenesis in a mouse model of KRAS-mutant human non-small cell lung cancer [34]. In a mouse model of pancreatic ductal adenocarcinoma, Fedele et al*.* found that KRAS inhibition via SHP2 inhibition inhibited tumor angiogenesis and vascularity [35]. In this study, we found that KRAS activation specifically in GA CSCs promotes expression of pro-angiogenic factors including VEGF-A, and that targeting both KRAS and VEGF-A in CSCs results in more-than-additive effects on primary tumor growth and metastasis.

The cancer stem cell theory proposes that CSCs play a key role in tumor initiation, progression, and metastasis. KRAS activation has been shown to contribute to the development and maintenance of CSCs in various tumor types, including gastric cancer. Additionally, VEGF-A has been implicated in the regulation of CSC self-renewal, differentiation, and promotion of angiogenesis. Thus, there is rationale to investigate the molecular mechanisms underlying the link between KRAS activation, VEGF-A expression, and CSCs. One study by Sennino B et al. found that inhibition of VEGF signaling by neutralizing antibodies or small molecule inhibitors significantly suppressed the growth of human pancreatic tumors with activating mutations in KRAS [36]. Another study by Majeti BK et al. showed that conditional deletion of VEGF in mouse models of KRAS-driven lung cancer significantly inhibited tumor growth and prolonged survival [37]. This study also showed that overexpression of VEGF in the lung epithelium of mice with KRAS mutations enhanced tumor growth and metastasis. These studies suggest that VEGF is indeed required for tumor progression driven by activated KRAS. One possible mechanism could involve the activation of downstream effectors of KRAS, such as the MAPK/ERK and PI3K/AKT pathways, which have been shown to regulate VEGF-A expression and angiogenesis [38]. Furthermore, the expression of various transcription factors, including HIF-1α and STAT3, may be regulated by KRAS and contribute to the transcriptional activation of VEGF-A [39]. In addition, other molecules such as miRNAs and exosomes, which have been implicated in the regulation of CSCs and angiogenesis, may also play a role in this mechanism. To further investigate the mechanistic link between KRAS activation, VEGF-A expression, and CSC behavior, future studies could focus on the identification of specific downstream effectors, transcription factors, and other molecules involved in this pathway. Additionally, the use of genetic and pharmacological approaches to modulate the activity of these molecules could provide insights into their functional roles in regulating CSC behavior and angiogenesis. Overall, understanding the mechanistic link between these pathways could lead to the development of novel therapeutic strategies targeting CSCs and angiogenesis in cancer.

To determine the translational relevance of the findings in this study to GA patients, we evaluated expression of the CSC marker CD44 and VEGF-A as prognostic factors for overall survival in a cohort of patients undergoing curative-intent gastrectomy for GA. CD44 and VEGF-A expression independently predicted worse overall survival. Our finding that patients with increased tumor levels of CD44 and VEGF-A expression had significantly worse overall survival after resection of their tumors suggests that this may be a subgroup in which combined KRAS inhibition and VEGF-A inhibition would be most beneficial.

Because RAS GTPases including KRAS have historically been difficult to target directly with drugs because of structure–function considerations [40], we inhibited the KRAS pathway using a MEK inhibitor. Several MEK inhibitors including trametinib, cobimetinib, and binimetinib are currently FDA-approved for use in patients with BRAF-mutated melanoma [41]. The MEK inhibitor used in this study, PD0325901, is currently being studied in clinical trials for patients with various solid tumors. There have been significant recent advances in the development of direct inhibitors of KRAS [42]. Sotorasib was developed as a direct inhibitor of KRAS^G12C^ (a common KRAS mutation). In a phase I trial of 59 patients with non-small cell lung cancer (NSCLC), 42 with colorectal cancer, and 28 with other solid tumors, sotorasib appeared to be well tolerated, with 11.6% of patients experiencing grade 3 or 4 toxicity [43]. Of the NSCLC patients, 32.2% had an objective response, with a total of 88.1% having disease control (objective response or stable disease). The median progression free survival (PFS) was 6.3months. In the colorectal cohort, 7.1% had a confirmed response with 73.8% having disease control, and a median PFS of 4months. Adagrasib is another potent, highly selective inhibitor of KRAS^G12C^. In a phase I/II study of 116 patients with pretreated NSCLC, the overall response rate to Adagrasib was 42.9%, disease control rate (DCR) was 79.5%, and median PFS was 6.5months (Spira et al*.* 2022 ASCO Annual Meeting). RMC-6236, developed by Revolution Medicine, directly targets multiple KRAS mutations at codon 12 and is currently being investigated in a phase I trial (Singh *M *et al*.* 2022 AACR Annual Meeting). Given that these agents that directly target oncogenic KRAS have few side effects, a combination strategy against oncogenic KRAS and VEGF-A as used in this study seems feasible in GA patients.

To the best of our knowledge, this is the first study to establish the importance of KRAS in GA CSCs in terms of promoting angiogenesis and metastasis and to demonstrate that inhibition of KRAS and VEGF-A may be an effective combination strategy. Studies were performed using human and mouse GA cell lines, in a genetically engineered, orthotopic implant, and two experimental metastasis mouse models. The relevance of these studies were confirmed by RNA protein analyses of patient tumors. These studies provide rationale for studying inhibitors of KRAS and VEGF-A in GA to block angiogenesis and metastasis.

## Supplementary Information

**Additional file 1:** **Supplemental Figure S1.** A-B. Graphs showing secreted angiogenic factors from AGS and MKN-45 grown as monolayers and as spheroids using the Proteome Profiler HumanAngiogenesis Array kit. C-D. Graphs showing secreted angiogenic factors from AGS and MKN-45 spheroid cells transduced with KRAS shRNA (sh.KRAS) or control scramble shRNA (sh.Scr). E. Western blot analysis for KRAS and VEGF-A in Tcon3077 organoid cells stably transduced with KRAS shRNA (sh.KRAS), VEGF-A shRNA (sh.VEGF-A) and/or control scramble shRNA (Original version in Supple Fig. S6A). F. Tube formation assay of MVECs or HUVECs in conditioned media from spheroids transduced with sh.KRAS and sh.Scr. Bars represent standard deviation. *p <0.05 compared to control.

**Additional file 2:** **Supplemental Figure S2.** A. A-B. IHC for CD44 and CD31 expression in mouse stomach tumors. C. Representative H&E photos of stomach tumors in mice sacrificed at 12 weeks.D. IVIS images after tail-vein injection of CD44(+) Tcon3077 cells transduced with sh.KRAS and/or sh.VEGF-A.

**Additional file 3:** **Supplemental Figure S3.** A. Photos of IVIS imaging and mouse footpad injected with Tcon3077 cells treated with KRAS shRNA (sh.KRAS) or control scramble shRNA (sh.Scr). B.Graph showing volume of lymph node metastases. Inset photo showing representative lymph nodes. C. Photos of H&E stain of representative lymph nodes, and IF staining for Lyve-1 (green) and CD44 (red). Graph showing the percent of cells positive for CD44 and Lyve-1. Bars represent standard deviation.*p <0.05 compared to control.

**Additional file 4:** **Supplemental Figure S4.** A. Heatmap of KRAS, VEGF-A, and CD44 based on the expression values from tumors and normal samples. B. Graph showing gene set enrichment analysis (GSEA) that compared the transcriptome data of the CD44 Low and CD44 High clusters using the MSigDB Hallmark genesets. C. Graph showing expression of KRAS and VEGF-A in gastric tumors, colored by the CD44 cluster (high, intermediate, or low). D. IF photos of tumors with high and low expression of CD44 (red), VEGF-A (green), and p-ERK1/2 (green). E-F. Kaplan–Meier overall survival curves stratified by expression of CD44 (E), and both CD44 and VEGF-A (F) in the FMUUH cohort.

**Additional file 5:** **Supplemental Figure S5.** A-B.These images are the original, unprocessed versions for western blots (Fig. 1C).C. These images are the original, unprocessed versions for western blots (Suppl. Fig. S1F).

**Additional file 6:** **Supplemental Figure S6.** A. These images are the original, unprocessed versions for western blots (Supple. Fig. S1E). B-C. These images are the original, unprocessed versions for western blots (Fig. 4A).  

**Additional file 7:** **Supplementary table 1.** Clinicopathological characteristics of FMUUH patients

## Data Availability

RNA-sequencing data is archived in Gene Expression Omnibus (GSE126304,https://www.ncbi.nlm.nih.gov/geo/query/acc.cgi?acc=GSE126304, token: wpaxeqkenlobhwr), and whole exome sequencing data in Sequence Read Archive (PRJNA521397, https://www.ncbi.nlm.nih.gov/sra/PRJNA521397) [14].

## References

[1] Wong MCS, Huang J, Chan PSF (2021). Global incidence and mortality of gastric cancer, 1980–2018. JAMA Netw Open.

[2] Wagner AD, Syn NL, Moehler M (2017). Chemotherapy for advanced gastric cancer. Cochrane Database Syst Rev.

[3] Comprehensive molecular characterization of gastric adenocarcinoma (2014). Nature.

[4] Samatar AA, Poulikakos PI (2014). Targeting RAS-ERK signalling in cancer: promises and challenges. Nat Rev Drug Discov.

[5] Till JE, Yoon C, Kim BJ (2017). Oncogenic KRAS and p53 loss drive gastric tumorigenesis in mice that can be attenuated by E-Cadherin expression. Cancer Res.

[6] Shimada S, Mimata A, Sekine M (2012). Synergistic tumour suppressor activity of E-cadherin and p53 in a conditional mouse model for metastatic diffuse-type gastric cancer. Gut.

[7] Yoon C, Till J, Cho SJ (2019). KRAS activation in gastric adenocarcinoma stimulates epithelial-to-mesenchymal transition to cancer stem-like cells and promotes metastasis. Mol Cancer Res.

[8] Kim MI, Kim SY, Lee JJ (2003). Prognostic effect of vascular endothelial growth factor and angiogenesis in gastric carcinoma. Cancer Res Treat.

[9] Park DJ, Thomas NJ, Yoon C, Yoon SS (2015). Vascular endothelial growth factor a inhibition in gastric cancer. Gastric Cancer.

[10] Wilke H, Muro K, Van Cutsem E (2014). Ramucirumab plus paclitaxel versus placebo plus paclitaxel in patients with previously treated advanced gastric or gastro-oesophageal junction adenocarcinoma (RAINBOW): a double-blind, randomised phase 3 trial. Lancet Oncol.

[11] Fuchs CS, Tomasek J, Yong CJ (2014). Ramucirumab monotherapy for previously treated advanced gastric or gastro-oesophageal junction adenocarcinoma (REGARD): an international, randomised, multicentre, placebo-controlled, phase 3 trial. Lancet.

[12] UKCCCR guidelines for the use of cell lines in cancer research. Br J Cancer 2000; 82: 1495–1509.10.1054/bjoc.1999.1169PMC236338310789715

[13] Vlachogiannis G, Hedayat S, Vatsiou A (2018). Patient-derived organoids model treatment response of metastatic gastrointestinal cancers. Science.

[14] Jun Y, Suh YS, Park S (2022). Comprehensive analysis of alternative splicing in gastric cancer identifies epithelial-mesenchymal transition subtypes associated with survival. Cancer Res.

[15] Gu Z, Eils R, Schlesner M (2016). Complex heatmaps reveal patterns and correlations in multidimensional genomic data. Bioinformatics.

[16] Subramanian A, Tamayo P, Mootha VK (2005). Gene set enrichment analysis: a knowledge-based approach for interpreting genome-wide expression profiles. Proc Natl Acad Sci U S A.

[17] Liberzon A, Subramanian A, Pinchback R (2011). Molecular signatures database (MSigDB) 3.0.. Bioinformatics.

[18] Yoon C, Park DJ, Schmidt B (2014). CD44 expression denotes a subpopulation of gastric cancer cells in which Hedgehog signaling promotes chemotherapy resistance. Clin Cancer Res.

[19] Prewett M, Huber J, Li Y (1999). Antivascular endothelial growth factor receptor (fetal liver kinase 1) monoclonal antibody inhibits tumor angiogenesis and growth of several mouse and human tumors. Cancer Res.

[20] Kelly KJ, Woo Y, Brader P (2008). Novel oncolytic agent GLV-1h68 is effective against malignant pleural mesothelioma. Hum Gene Ther.

[21] Jackson DG (2019). Hyaluronan in the lymphatics: the key role of the hyaluronan receptor LYVE-1 in leucocyte trafficking. Matrix Biol.

[22] Cristescu R, Lee J, Nebozhyn M (2015). Molecular analysis of gastric cancer identifies subtypes associated with distinct clinical outcomes. Nat Med.

[23] Lin JX, Yoon C, Li P (2021). Increased CD44 expression and mek activity predict worse prognosis in gastric adenocarcinoma patients undergoing gastrectomy. J Gastrointest Surg.

[24] Alison MR, Lin WR, Lim SM, Nicholson LJ (2012). Cancer stem cells: in the line of fire. Cancer Treat Rev.

[25] Ye X, Weinberg RA (2015). Epithelial-mesenchymal plasticity: a central regulator of cancer progression. Trends Cell Biol.

[26] Shibue T, Weinberg RA (2017). EMT, CSCs, and drug resistance: the mechanistic link and clinical implications. Nat Rev Clin Oncol.

[27] Voon DC, Wang H, Koo JK (2013). EMT-induced stemness and tumorigenicity are fueled by the EGFR/Ras pathway. PLoS ONE.

[28] Min J, Vega PN, Engevik AC (2019). Heterogeneity and dynamics of active Kras-induced dysplastic lineages from mouse corpus stomach. Nat Commun.

[29] Chippalkatti R, Abankwa D (2021). Promotion of cancer cell stemness by Ras. Biochem Soc Trans.

[30] Blaj C, Schmidt EM, Lamprecht S (2017). Oncogenic effects of high MAPK activity in colorectal cancer mark progenitor cells and persist irrespective of RAS mutations. Cancer Res.

[31] Moon BS, Jeong WJ, Park J (2014). Role of oncogenic K-Ras in cancer stem cell activation by aberrant Wnt/beta-catenin signaling. J Natl Cancer Inst.

[32] Okada M, Shibuya K, Sato A (2014). Targeting the K-Ras–JNK axis eliminates cancer stem-like cells and prevents pancreatic tumor formation. Oncotarget.

[33] Yuan XH, Yang J, Wang XY (2018). Association between EGFR/KRAS mutation and expression of VEGFA, VEGFR and VEGFR2 in lung adenocarcinoma. Oncol Lett.

[34] Takahashi O, Komaki R, Smith PD (2012). Combined MEK and VEGFR inhibition in orthotopic human lung cancer models results in enhanced inhibition of tumor angiogenesis, growth, and metastasis. Clin Cancer Res.

[35] Coley AB, Ward A, Keeton AB (2022). Pan-RAS inhibitors: hitting multiple RAS isozymes with one stone. Adv Cancer Res.

[36] Sennino B, Ishiguro-Oonuma T, Wei Y (2012). Suppression of tumor invasion and metastasis by concurrent inhibition of c-Met and VEGF signaling in pancreatic neuroendocrine tumors. Cancer Discov.

[37] Majeti BK, Lee JH, Simmons BH, Shojaei F (2013). VEGF is an important mediator of tumor angiogenesis in malignant lesions in a genetically engineered mouse model of lung adenocarcinoma. BMC Cancer.

[38] Shibuya M (2011). Vascular Endothelial Growth Factor (VEGF) and its receptor (VEGFR) signaling in angiogenesis: a crucial target for anti- and pro-angiogenic therapies. Genes Cancer.

[39] Lv X, Li J, Zhang C (2017). The role of hypoxia-inducible factors in tumor angiogenesis and cell metabolism. Genes Dis.

[40] Cox AD, Fesik SW, Kimmelman AC (2014). Drugging the undruggable RAS: mission possible?. Nat Rev Drug Discov.

[41] Zhao Y, Adjei AA (2014). The clinical development of MEK inhibitors. Nat Rev Clin Oncol.

[42] Conroy M, Cowzer D, Kolch W, Duffy AG (2021). Emerging RAS-directed therapies for cancer. Cancer Drug Resist.

[43] Hong DS, Fakih MG, Strickler JH (2020). KRAS(G12C) inhibition with sotorasib in advanced solid tumors. N Engl J Med.

